# Fermented Carrot Pulp Regulates the Dysfunction of Murine Intestinal Microbiota

**DOI:** 10.1155/2022/2479956

**Published:** 2022-03-16

**Authors:** Chenchen YU, Ying Liu, Zhang Xuemei, Aijin Ma, Tan Jianxin, Tian Yiling

**Affiliations:** ^1^College of Food Science and Technology, Hebei Agricultural University, Baoding Hebei, China; ^2^College of Forestry, Hebei Agricultural University, Baoding Hebei, China; ^3^School of Food and Health, Beijing Technology and Business University, Beijing, China

## Abstract

It was the focus of attention that probiotic control drink was packed with prebiotic nutrients and lactic acid bacteria. So, this study is aimed at revealing that the fermented carrot pulp regulation and protection function to the intestinal microecological disorders usually induced by antibiotic treatment. First, we study on lactobacillus fermentation conditions and effects on the secondary metabolism of fermented carrot juice, get its phenolic acids up, and get its flavonoids down. Then, establishment of the dysbacteriosis mouse model was used to validate the fermented carrot pulp prevention and treatment of intestinal microbiota imbalance. After the antibiotic treatment, the mice showed impotence, laziness, slow movement, weight loss, thin feces, dull hair, and anal redness, while the mice in the control group were all normal in terms of the mental state, diet, weight, and bowl movement. Along with the treatment, the abnormal conditions of the mice in the model group and natural recovery group improved in different degrees, indicating that the fermentation treatment is of help to the intestinal microbiota recovery. The fermentation-treated group of mice recovered close to normal that the diarrhea disappeared, and the weight gain, mental state, and the feces became normal. The serum antioxidant (SOD, GSH, and MDA) levels of the mice were checked. The superoxide dismutase (SOD) levels and glutathione (GSH) levels in the ordinary fermentation-treated group and probiotic fermentation-treated group were significantly increased compare to the natural recovery group. The malondialdehyde (MDA) levels showed great differences between the fermentation-treated groups and the blank group. At last, the 16sRNA analysis revealed that the microbiota richness and diversity in probiotic fermentation (J) are much higher than those in the model group (H), ordinary fermentation group (I), and blank group (G). Groups J and I are of significantly higher antioxidant level than group H; however, only the glutathione (GSH) level in group J increased dramatically but not those in the other three groups. Antibiotic treatment-induced mouse intestinal microecological disorder reduce the microbiota richness and diversity. Prebiotics fermented carrot pulp treatment can help in the recovery from the microbiota richness and diversity level prior to the antibiotic treatment, which suggests it can regulate and protect the murine intestinal microbiome.

## 1. Introduction

Carrot (*Daucus carota L.*) is an herb of dicotyledonous family Umbelliferae, also known as red root, golden bamboo shoots, clove radish, and the root of the umbelliferous plant carrot. Carrot is an ordinary vegetable or used as animal food traditionally, not making full use of the carrot from both the nutrition and economy point of view. The consumption of carrots in the long run has many effects in promoting human health such as antioxidant and antiaging effects, development and growth promotion, vision protection, skin health, cancer prevention, chemotherapy side effects reduction, immunity improvement, intestinal micro ecology protection, appetite increasing, and digestion promotion [1–7]. In summary, carrot is a vegetable with rich nutrients and excellent functional ingredients.

Making carrot juice, which is obtained by crushing fresh carrots, is the main processing method in the food processing industry. It is very close to the fresh raw carrot in flavor and nutrition, thus good to health. At present, the research on carrot juice is focused on the juice made by carrot only or the composite fruit and vegetable juice that is rich in functional factors [8].

Lactic acid bacteria (LAB) are Gram-positive, non-spore-forming cocci, coccobacilli, or rods [9, 10]. As one of the probiotics beneficial to human health, lactic acid bacteria can improve the food flavor, protect and regulate the balance of the intestinal microbiota, promote the gastrointestinal motility and nutrients absorption, decrease the cholesterol level, prevent and against cancer, and enhance the immunity [11–13]. Thus, lactic acid bacteria research from different perspectives brought promising insights in benefiting human health, in which the host microecology regulation studies rooted in that lactic acid bacteria can adhere to the intestines and produce organic acids such as lactic acid and acetic acid to inhibit the pathogenic bacteria growth and reproduction and, therefore, maintain the balance of the intestinal ecological microbiota [14, 15].

Probiotic-fermented carrot juice is a recently developed beverage that is nutrition enriched, flavor pleasant, and good to human health, thus welcomed by increasing consumers. The probiotic fermentation can specifically diminish the medicinal astringency and the grassy scent, which has been confirmed by many studies: Demi et al. fermented carrot juice with *Lactobacillus RSKK1602*; Bergqvist et al. fermented carrot juice via two methods using two types of carrot juice with *Lactobacillus pentosus FSC1* and *Leuconostoc FSC2* separately, through which they confirmed that the fermentation can improve the iron utilization in carrot juice; Cliff et al. developed a new type of lactic acid-fermented carrot juice milk with different carrot juice proportions, different yogurt viscosities, and different fermentation strains [16–18].

The intestines are the largest digestive and excretory organ, where there are live and more than 100 trillion bacteria that form the intestinal microecological system [19]. There are at least 4 × 1013 colonized microbial cells and more that 10 million microbial genes in human gut [20–22]. The types and counts of the intestinal microbiota are relatively stable and interactively live together to keep the microecological balance and the health of the host. It has been proven that imbalance of the microbiota equilibrium will cause various disorders [23] including lipopolysaccharide absorption and intestinal permeability, inflammatory response, insulin resistance, and metabolic disorders, which in turn induce metabolic syndrome (MS), which can further distort the intestinal microbiota. The formation of a vicious circle may also induce or aggravate liver damage [24]. Therefore, the stability of the intestinal microbiota is particularly important for human health. Recently, studies showed the effect of secondary metabolite (such as flavone, triterpene, and alkaloid) and metal-ion (Zn) on the intestinal microorganism of living organisms to improve body health [25–28].

Since the golden age of the antibiotic development and utilization at the 1950s to 1970s, antibiotic has brought advantages to human, while also bringing negative effects, such as gastrointestinal reactions, dysbacteriosis, and pathogen amplification, which further adversely affected the animals' health and nutrition absorption [25, 29–31]. Abuse of antibiotics, including the prophylactic usage, will damage the body [32–34].

Fermented carrot pulp combines fruits, vegetables and lactic acid bacteria with pleasant flavor and rich nutrition. It can be used for the microecological disorder treatment, without the side effect of the medical treatment. Economically, the fermentation processing increased the added value of the raw materials of fruits and vegetables.

The use of probiotics in the deep food processing of fruits and vegetables has been limited to the kimchi production. With the food science and technology development, probiotic fermentation has been applied in the fruit and vegetable beverage production. It is worth noting that the current research on fermented carrot pulp is still in its infancy, and there are still many problems that need to be explored and solved. First, the active lactic acid bacteria are stable at a certain temperature, so the strain activity tends to be reduced or even inactivated in transportation, storage, and sales, directly affecting the shelf life. Therefore, the discovery and development of a special strain with great fruit and vegetable fermentation characteristic is crucial for the industry. Secondly, the standards and the safety criteria of the fruit and vegetable fermentation remain to be satisfied. Finally, it is critical to improve the stability of the fermented fruit and vegetable products, speed up the research and development of functional probiotic fruit and vegetable foods, and vigorously promote the industrialization.

## 2. Materials, Instruments, and Methods

### 2.1. Animals

All experiments were carried out with Hebei Agricultural University ethical approval and a China Laboratory Animal Quality control of Reproductive and Development (GB/T39647, 2020). 42 Kunming mice (male, 18~22 g, SPF grade) from Beijing Weitong Lihua Experimental Animal Technology Co. Ltd. And they were housed under normal laboratory conditions (12 h light dark cycle, lights on at 7 a.m., 21 ± 1°C, humidity 50 ± 5%). Mice were adapted in the laboratory for a week before the procedures. Then, the mice were randomly separated into four groups, namely, blank group (KB), model group (MX), ordinary fermentation group (EI1), and probiotic fermentation group (EI2).

### 2.2. Reagents and Instruments

Ordinarily fermented and rebiotics-fermented carrot pulps are used [35]. Ampicillin sodium (0.5 g/mL) is from Shanghai Shenggong Bioengineering Co. Ltd. Total cholesterol (TC) test kit, triglyceride (TG) test kit, malondialdehyde (MDA) test kit, superoxide dismutase (SOD) test kit, and reduced glutathione (GSH) test kit are from Nanjing Jiancheng Bioengineering Institute.

Electronic analysis balance is obtained from Yuyao Jinnuo Tianping Instrument Co., Ltd.; Pipette from Shanghai Thermo Fisher Scientific Instrument Co. Ltd.; Ultra-low temperature refrigerator from SANYO (Japan); and 1500-823 microplate reader from Thermo Fisher Scientific.

### 2.3. Methods

#### 2.3.1. Fermented Carrot Juice

Carrot juice was prepared from fresh carrots using a juicer and pasteurizing the juice at 85°C for 30 min. With sterilized carrot juice as raw material, fermented juice was produced via a liquid-solid fermentation method.

#### 2.3.2. Detection the Contents of Total Polyphenol in Carrot

The total polyphenol content of carrot juice (including fermented juice) was determined by Folin-Ciocalteu assay. 15 *μ*L of carrot juice was mixed with 2.5 mL of 0.2 N Folin-Ciocalteu reagent for 5 min, and then, 2.0 mL of 75 g/L Na_2_CO_3_ solution was added. The total polyphenol content was expressed as *μ*g gallic acid equivalent per milliliter using the calibration curve of gallic acid (0–2000 *μ*g/mL). The working curve of aba copter in I was as follows: *A* = 0.0071*x* − 0.0084 (*R*^2^ = 0.9990).

#### 2.3.3. Measurement of Total Flavonoids

The total flavonoid was determined using the NaNO_2_-Al(NO_3_)_3_-NaOH colorimetric method with a slight modification (Muhamad, Muhmed, Yusoff, & Gimbun, 2014). 200 *μ*L of sample solution and 400 *μ*L of 0.066 mol/L NaNO_2_ were mixed fully in a centrifuge tube and kept for 5 min. Then, 60 *μ*L of 10% (*w*/*v*) AlCl_3_ was added to the centrifuge tube. Six minutes later, 400 *μ*L of 1 mol/L NaOH was put into the tube. The absorbance wavelength and reference were 510 nm and rutin, respectively. The working curve of aba copter in I was as follows: *A* = 1.17*X* + 0.01 (*R*^2^ = 0.9994).

#### 2.3.4. Establishment of the Dysbacteriosis Mouse Model

The 31 mice (experimental groups MX, EI1, and EI2) were intragastrically administered with ampicillin (125 mg/mL, 2.5 mg/g body weight) twice a day for 4 days. The 11 blank mice (KB) were given a similar volume of sterile water. Multiple measurements were observed and recorded daily during the model building including the behavior of the mice, hair, fecal characteristics, and diarrhea. After the model building, one mouse from each group (from the experimental group) was randomly selected for the feces collection, and then the mice were killed and dissected for the cecum observation (see Figure 1(a)). In the intestinal microbiological analysis results, the MX1 represents the treated mice that were sacrificed prior to the treatment and KB1 represents the control mouse.

#### 2.3.5. Regrouping and Treatment

The 30 antibiotic-treated mice were separated into three groups randomly for a 21-day treatment: model group (MX2), ordinary fermentation groups (EI1, EII1), and probiotic fermentation groups (EI2, EII2). The ordinary fermentation group and probiotic fermentation group were gavages fermented products on 0.2 mL/10 g body weight, and the MX2 control group mice were given similar amount of sterile water.

#### 2.3.6. Observation of the Mice

The mice were monitored every day after the treatment. The behavior, hair, activity, feces, and body weight were recorded. The feces were collected 2 hours after the gavaging.

#### 2.3.7. Other Indicators

Mice were fasted for 16 hours after the last day treatment; then, the body weight was measured, and the feces and the blood were collected. The blood samples were placed in a 1.5 mL centrifuge tube for 1 hour, then centrifuged for 10 minutes at 3500 rpm/min to collect the serum. Afterwards, the TC, TG, MDA, SOD, and GSH levels were tested.

#### 2.3.8. Intestinal Microbiota Analysis

Through DNA extraction and detection, PCR amplification, product purification, library preparation, and detection and through the process of computer sequencing by Miseq, the diversity of bacteria was sequenced.

#### 2.3.9. Statistics and Data Processing

All the samples were processed and analyzed in quintuplicate. The values were expressed as the means ± SD. Statistical analyses were performed using IBM SPSS Statistics version 17.0 (SPSS Inc., Chicago, IL, USA). One-way analysis of variance (ANOVA) followed by Student's *t*-test was applied to determine the statistical significance of differences between data. Differences with *P* < 0.05 were considered statistically significant. Bcl2fastq (v2.17.1.14) image processing software was used for base pair identification, and Cutadapt (v1.9.1), Vsearch (1.9.6), and Qiime (1.9.1) were used for the sequencing data optimization, OTI cluster analysis, species annotation, and counting and R packages for visualization.

## 3. Results

### 3.1. Effect on Polyphenol and Flavonoids in Fermentation

Carrot flavor and secondary metabolites have been different between before and after fermentation, such as about 13% fewer flavonoids, while polyphenol content increases 38.01% (see Table 1). In fact, flavonoid uptake in the small intestine is relatively low, suggesting the absorption (including absorbed and combined) processing of them will reach the large intestine and contact with the microflora of the colon [26]. Now, flavonoids might be catalyzed to phenolic acid by fermentation, that is comparable with conjugates by colonic microorganisms, and there are enhanced absorption and utilization efficiency.

### 3.2. Verification of the Dysbacteriosis Mouse Model

We investigated the intestinal microbiota relative abundance through 16sRNA analysis. We found that the genera Polymorphic bacillus, Prevos, Pleurotus, Alistipes, Parasutterella, Lactobacillus, and Rosella were much less abundant compare to the control group (KB1), while the cerevisiae, Enterococcus, and Robinsoniella are much higher in the dysbacteriosis mouse model than the control group (KB1) (Figure 1(b)).

Meanwhile, there were Klebsiella and Enterococcus, which are highly pathogenic to human and were detected within MX1. Therefore, the reduction or disappearance of the bacillus that are beneficial to human and the increase of the cocci that are pathogenic to human suggested the imbalance of the intestinal microbiota from the antibiotic treatment [36, 37].

We further did the anatomy analysis for the mice KB1 and MX1 and found that the cecal wall of the MX1 is thinned, 2-4 times swelled compare to the KB1, and the contents were watery, which is obviously differentiated from the control mouse. These changes suggested that intragastric administration of ampicillin is an effective way of establishing a dysbacteriological mouse model.

### 3.3. Mouse Weight Changes

The weight of all the mice is comparable prior to the model building, while it showed significant difference after the model building (Table 2, 1 w), and later recovered to the similar level after the model group or treatment (Table 2, 4 w). We can also see that the original fermentation and probiotic fermentation-treated mice are of speedy recovery in terms of weight gaining comparing to the model group indicating that the fermentation treatments are of the function that can help the intestinal microbiota reestablish faster.

### 3.4. Other Factor Change for the Mice

All the mice were in very similar normal condition prior to the model building. After the antibiotic treatment, the mice showed impotence, laziness, slow movement, weight loss, thin feces, dull hair, and anal redness, while the mice in the control group were all normal in terms of the mental state, diet, weight, and bowel movement. Along with the treatment, the abnormal conditions of the mice in the model group and natural recovery group improved in different degrees, indicating that the fermentation treatment is of help to the intestinal microbiota recovery. The fermentation-treated group of mice recovered close to normal that the diarrhea disappeared, and the weight gain, mental state, and the feces became normal. In the natural recovery group, the diarrhea of the mice was alleviated, the hair gradually returned to the luster but slightly yellow, and the stool color became lighter [38]. The status of each group before, during and after the model building, is sown in Table 3.

### 3.5. The SOD, GSH, and MDA Levels in the Mouse Serum

We also checked the effect of each fermentation broth on the serum antioxidant (SOD, GSH, and MDA) levels of the mice. The tested results and significant levels between different groups calculated by test are shown in Table 4. We can see that the superoxide dismutase (SOD) levels and glutathione (GSH) levels in the ordinary fermentation-treated group and probiotic fermentation-treated group were significantly increased compared to the model. The malondialdehyde (MDA) levels showed great differences between the fermentation-treated groups and the model group and significantly reduced. Oxidation system regulates the NF-*κ*B and MAPK signaling pathways and ultimately maintains the intestinal health of animal bodies [28].

### 3.6. TC and TG in the Mouse Serum

TC and TG in the serum are closely related to lipid metabolism in the body. In order to illustrate if the fermentation broth treatment to the mouse model will influence the lipid metabolism, we tested the TC and TG in the mouse serum from all the groups as shown in Table 5. We can see that the TC and TG show no difference between the treated group and the control group indicating that the fermentation broth treatments did not affect the lipid metabolism.

### 3.7. Microbial Diversity Analysis of the Mouse Feces

#### 3.7.1. OTU Analysis

OTU analysis refers to the unified mark artificially set for a taxon (genus, species, grouping, etc.) for the convenience of analysis in population genetics research. Sequences are usually divided into different OTUs based on a 97% similarity threshold, each of which is usually treated as a microbial species. If the similarity is less than 97%, it can be considered belonging to different species; if the similarity is less than 93-95%, it can be considered belonging to different genera.

We did the OTU analysis to evaluate the microbial diversity for the dysbacteriosis mouse model after treatment. The ordinary fermentation groups EI1 and EII1 and the probiotic fermentation groups EI1 and EII2 were grouped together to calculate the average. The OTU results are shown in Table 6 and indicate that the abundance of the intestinal microbiota in the mice after treatment with carrot fermentation broth (170 and 167) is higher that of the natural recovery group (157) and the control group (156).

We further checked the type of the microbiota in the four groups as indicated in Figure 2. The type of the microbiota in the four groups is largely the same (Figure 2(a)), which suggested that the carrot fermentation broth gavaging can bring the total intestinal microbiota level back to the normal level prior to the antibiotic treatment. In terms of the bacterial types, we first ranked all of the bacterial strains detected from the OTU analysis, the top 30 are mostly bacilli and pseudobacteria, and abundance of the strains was displayed through heatmap (Figure 2(b)).

The microbiota type and abundance analysis suggested that after the antibiotic treatment, the intestinal microbiota is dysfunctional indicated by the bacillus abundance reduction and cocci abundance, and the harmful microorganisms increase. After 21 days of continuous fermented carrot pulp administration or natural recovery, the intestinal microbiota from all of the mice have been improved and repaired to varying degrees. Among the top 30 abundant strains, OTU17, a probiotic, plays an important role in metabolism regulation, obesity, and tumor controlling and is enriched in the probiotic-fermented group. OTU9, a Lactobacillus, and OTU15, a lactic acid bacterium Lactobacillus genus, are essential microbiota in the human intestine and maintain the ecological balance of the intestinal microbiota. Their abundances are higher in the probiotic fermentation group than in the ordinary fermentation group, indicating that lactobacillus can colonize in the intestines with the probiotic assistant. OTU18 Rosporia can be used in obesity prevention and treatment, OTU12 is a fecal sterol-producing bacterium and can decompose cholesterol, in which abundance is higher in the fermented carrot pulp-treated mice, especially the probiotic-fermented pulp-treated mice than the model group and control groups. In summary, the OTU analysis result inferred that fermented carrot pulp treatment can bring back the microbiota back to the similar level before antibiotic treatment, and the probiotic fermented pulp treatment can help the certain beneficial bacteria colonization compared to the ordinary fermented pulp.

#### 3.7.2. Alpha Diversity Analysis

Alpha diversity analysis is aimed at studying the diversity within a single sample, which represents the number of species in the microbial community and predicts the abundance and diversity of environmental colonies with a series of statistical indices including ACE index, Chao index, Shannon index, Simpson index, and Good's Coverage index.

The ACE index of the model group is close but lower than that of ordinary fermentation group; the Chao1 index of the natural recovery group is slightly higher than that of the ordinary fermentation group and the probiotic fermentation group (Table 7), indicating that the colony diversity of natural recovery group and ordinary fermentation group was higher than that of probiotic fermentation group. The Shannon and the Simpson index are higher in the probiotic fermentation group than in the natural recovery group (Table 7), indicating that the colony diversity of the probiotic fermentation and the ordinary fermentation group was superior to that of the natural recovery group. Good's Coverage index was 1 in every tested groups (Table 7), indicating a high bacterial coverage in the tested mouse models.

#### 3.7.3. Beta Diversity Analysis

The beta diversity index was used to measure the diversity differences among samples. Beta diversity analysis used heatmap to intuitively represent the diversity matrix (Figure 3).

The UniFrac index is used to illustrate the differences of species communities between samples, which is positively correlated with the difference of samples. We calculated the weighted UniFrac (Figure 3(a)) and unweighted UniFrac (Figure 3(b)), where the weighted UniFrac is considering the sequence/species abundance. The beta diversity analysis in Figure 3 indicated that there is week clustering among these microbiota from the mouse model. In order to further reveal the diversity differences, we employed Principle Component Analysis.

Principle Component Analysis (PCA) is used for predicting the differences in sample diversity and to how much degree the differences are between samples. The distance between the samples indicates positively the similarity of the microbial aggregation in the samples. As shown in Figure 4(a), for the PC1-PC2 analysis, KB2, EI2, and EII2 are close, thus similar to each other, while EI1 and EII1 are different to each other since there they were separated; and MX2 is of a relatively large difference with all the other samples as it locates at the negative axis of PC1-PC2. Likewise, in the PC1-PC3 (Figure 4(b)) and PC2-PC3 (Figure 4(c)) analysis, KB2, EI2, and EII2 are close and similar to each other, EI1 is different with EII1, and MX2 is different with the other testing groups. In summary, we can conclude from the PCA analysis that the intestinal microbiota of the probiotic fermentation-treated mouse were recovered to the level of the natural recovery; therefore, probiotic fermentation is of regulation and improvement effect on the intestinal microbiota balance.

#### 3.7.4. Microbiota Diversity Classified by Phylum

The species diversity of the samples indicated that there are eight phyla from all the samples: *Bacteroidetes*, *Proteobacteria*, *Firmicutes*, *Verrucomicrobia*, *Saccharibacteria*, *Actinobacteria*, *Tenericutes*, and *Deferribacteres*. As shown in phylum analysis in Figure 5, *Bacteroidetes* abundance takes the largest proportion in most of the samples; moreover, its proportion in probiotic fermentation group is higher than that in the control group, the model group, and the ordinary fermentation group, indicating that the prebiotics are more conducive to the species diversity of the *Bacteroidetes.* Another significant change of the phylum is the *Proteobacteria* proportion in the control group is dominant, while the rest of the groups are rare. This *Proteobacteria* dramatic decrease indicates that *Proteobacteria* is affected heavily by the antibiotic and hard to resume after the mouse model building and recovery. The proportion of *Firmicutes* was second to that of *Bacteroidetes*, and the abundance in the probiotic fermentation group was over 5 times higher than those of other groups, indicating that ordinary fermentation is more conducive to the growth and colonization of the *Firmicutes. Verrucomicrobia* was not detected from the control group, while it was detected within the model group and fermentation-treated groups. Although *Actinobacteria* can be detected from every group, the proportion is relatively low.

#### 3.7.5. Microbiota Diversity Classified by Genus

We identified 44 genera from all the samples that include *Bacteroides*, *Prevotellaceae_UCG-001*, *Akkermansia*, *Lachnospiraceae_NK4A136_group*, *Lachnospiraceae_UCG-001*, *Alloprevotella*, and *Alistipes*. The 30 most abundant genus proportions in each sample are shown in Figure 6. The microbiota genus in the control group was *Bacteroides*, *Prevotellaceae_UCG-001*, *Alloprevotella*, *Alistipes*, *Parasutterella*, and *Candidatus_Saccharimonas*. Samples from treated mouse models include *Bacteroides*, *Prevotellaceae_UCG-001*, *Akkermansia*, *Lachnospiraceae_NK4A136_group*, *Lachnoclostridium*, and *Alistipes*. The ordinary fermentation group mainly included *Bacteroides*, *Prevotellaceae_UCG-001*, *Lachnospiraceae*, *Lachnospiraceae_NK4A136_group*, Ruminococcaceae_UCG-014, and Rosella. The probiotic fermentation group samples mainly included *Bacteroides*, *Prevotellaceae_UCG-001*, *Alloprevotella*, *Candidatus_Saccharimonas*, *Alistipes*, and *Parasutterella*. The colony level of the probiotic fermentation was consistent with that of the control group. There were three types of genera in the model group which were consistent with those in the control group and two types of genera in the ordinary fermentation group which were consistent with the control group, indicating that the colony level recovered to the control level after the probiotic fermentation pulps treatment.

## 4. Conclusion

As a new type of fermented beverage, fermented carrot pulp can effectively improve and regulate the intestinal microbiota and maintain the balance of the microbiome. Moreover, compared with the treatment of intestinal microbiota imbalance from drugs, fermentation carrot juice with the addition of probiotics is more acceptable in flavor and taste.

In summary, our study shows that fermented carrot pulp can regulate and protect the intestinal microbiota and thus can be used as a regulator of intestinal microecology for the prevention and treatment of intestinal microbiota imbalance. There are also foods with different tastes that provide a new reference for microecological disorders, which provide important significance for the limitations of drug-mediated microecology.

## Figures and Tables

**Figure 1:** (a) Validation of the dysbacteriosis mouse model. (b) Mouse anatomy analysis. The cecal wall of the MX1 is thinned, 2-4 times swelled compare to the KB1, and the contents were watery.

**Figure 2:** (a) Venn diagram of the strain types from OUT analysis (G and H: model group, I: fermentation group, J: probiotic fermentation group). (b) Heatmap diagram of the top 30 strains abundance in OUT result. OTU44 is *Bacillus*, OTU11 is *Pseudomonas*, OTU22 is *Alcaligenes*, OTU10 is *Bacteroides* and *Klebsiella*, OTU12 is a *fecal sterol-producing bacterium*, OTU9 is *Lactobacillus*, OTU15 is *Lactobacillus genus*, OTU26 is *Helicobacter*, OTU18 is *Rosporia*, OTU6 is *polymorphic rod*, OTU14 is *Helicobacter Bacillus*, and OTU45, 30, 1, 3, 4, 7, 8, 74, 17, 21, 16, 102, 37, 24, and 19 are *Bacteroides.*

**Figure 3:** Heatmap diagram of beta diversity.

**Figure 4:** Principle Component Analysis (PCA).

**Figure 5:** Phylum analysis.

**Figure 6:** Genus analysis.

**Table 1:** Effect on polyphenol and flavonoids in fermented carrot.

Component	Carrot puree	Fermented juice	Variation (%)
Total polyphenol (mg/100 g)	29.54 ± 0.0033	67.55 ± 0.0007	+38.01
Total flavonoids (mg/mL)	0.19 ± 0.0609	0.06 ± 0.0005	-0.13

**Table 2:** The weight change of mice in different experimental groups ($\bar{x}\pm s$, g).

Group	3 d (before molding)	1 w	2 w	3 w	4 w
Blank	20.16 ± 0.42	31.25 ± 3.44	38.80 ± 2.37	44.21 ± 1.61	48.18 ± 1.20
Model	20.14 ± 0.38	28.33 ± 2.19^b^	34.84 ± 1.87^b^	40.76 ± 1.14^b^	45.20 ± 1.71
Fermentation	—	27.19 ± 2.39^b^	34.59 ± 1.46^b^	42.79 ± 1.43	45.41 ± 1.77
Probiotic fermentation	—	28.58 ± 2.00^b^	35.64 ± 1.51^b^	42.90 ± 1.61	45.80 ± 0.97

^a^ *P* < 0.01; ^b^*P* < 0.05.

**Table 3:** General condition changes in mice.

	Group	Weight increased	Mental state	Hair	Feces
Before molding	All	Normal	Normal	Smooth-coated	Dry, brown-black
Molding	Blank	Normal	Normal	Normal	Normal
	Model	Slow	Dispirited	Lusterless, yellowing	Diarrhea
Treatment	Blank	Normal	Normal	Normal	Normal
	Model	Slow	In-normal	Luster, yellowing	Diarrhea relief
	Fermentation	Normal	Normal	Luster	Diarrhea abated
	Probiotic fermentation	Normal	Normal	Luster	Diarrhea abated

**Table 4:** The effect of fermentation liquor on antioxidant levels in serum of mice ($\bar{x}\pm s$).

Group	SOD (U/mg)	GSH (*μ*mol/g)	MDA (nmol/mg)
Blank	172.39 ± 23.16^b^	30.85 ± 7.53^d^	18.38 ± 11.04^d^
Model	132.19 ± 12.90	16.84 ± 6.83	31.04 ± 19.06
Fermentation	161.76 ± 10.11^c^	23.99 ± 5.68^d^	11.82 ± 6.06^d^
Probiotic fermentation	154.80 ± 12.40^c^	16.47 ± 3.39^af^	10.13 ± 1.68^d^

Compared with the blank group, ^a^*P* < 0.01 and ^b^*P* < 0.05. Compared with the model group, ^c^*P* < 0.01 and ^d^*P* < 0.05. In comparison between experimental groups, ^e^*P* < 0.01 and ^f^*P* < 0.05.

**Table 5:** Effects of fermented liquid tablets on serum lipid levels in sera of mice ($\bar{x}\pm s$).

Group	TC (*μ*mol/g)	TG (mmol/g)
Blank	4.30 ± 0.79	2.32 ± 0.56
Model	4.18 ± 0.77	2.35 ± 0.48
Fermentation	3.54 ± 0.71	2.02 ± 0.78
Probiotic fermentation	4.59 ± 0.88	2.13 ± 0.42

Compared with the blank group, ^a^*P* < 0.01 and ^b^*P* < 0.05.

**Table 6:** The result of OTU.

Sample	Blank	Model	Fermentation	Probiotic fermentation
OTU	156	157	170	167

**Table 7:** The result of alpha analysis.

Group	Sample	ACE	Chao1	Shannon	Simpson	Good's Coverage
Blank	KB2	147.362	162.2	4.342	0.864	1
Model	MX2	162.396	167	4.981	0.819	1
Fermentation	EI1	157.549	158.875	4.086	0.843	1
—	EII1	157.876	156.6	4.357	0.895	1
Probiotic fermentation	EI2	146.382	144.125	4.742	0.94	1
—	EII2	139.563	139	4.567	0.927	1

## Data Availability

The data used to support the findings of this study are included within the article.
